The article "Analysis of Erhu Performance Effect in Public Health Music Works Based on Artificial Intelligence Technology" was retracted in 2023. Reasons: signs of a paper mill; suspected computer-generated content; unreliable results or conclusions; concerns about the data.

# Analysis of Erhu Performance Effect in Public Health Music Works Based on Artificial Intelligence Technology

**DOI:** 10.1155/2022/9251793

**Published:** 2022-09-01

**Authors:** Li Yang

**Affiliations:** Music Department, Normal College, Changshu Institute of Technology, Changshu 215500, China

## Abstract

With the rise of Erhu teaching in recent years, a large number of people have joined the team to learn Erhu playing. However, due to the high cost of teaching and the unique one-to-one teaching mode between teachers and students, Erhu education resources are very scarce. Learning Erhu performance has become a luxury activity. Nowadays, with the rise of artificial intelligence, computer music is developing rapidly. Music has two important aspects: composition and performance. Different kinds of instruments convey different styles, and players inject different rhythms and dynamics into their performance, thus producing rich expressive force. The development of image style conversion, which opens people's evaluation of music performance, is an important issue in many fields of artificial intelligence (it is also known as intelligence, machine intelligence, referring to the intelligence shown by the machine made by people. Usually, artificial intelligence refers to the technique of presenting human intelligence through ordinary computer programs). For an Erhu song, there are various factors that affect its effectiveness, and there are many indexes to evaluate it, such as sense of rhythm, expressive force, musical sense, style, and so on. Using a computer to simulate the evaluation process is essential to find out the mathematical relationship between the factors that affect the performance of music and the evaluation indexes. Neural network is a kind of mathematical model proposed by simulating the way of thinking of human brain in artificial intelligence. It has the advantages of not having strict requirements on data distribution, nonlinear data processing method, strong robustness, and dynamics and is very suitable for the mathematical model of evaluation system. In addition, the neural network also has a strong theoretical basis, and their application in various industries has developed basically mature. This paper tries to introduce a deep neural network mathematical model into the evaluation system of Erhu performance, and the experimental results prove the reliability and practicality of the method in this paper. It can provide a method basis and theoretical reference for evaluation of Erhu performance effect.

## 1. Introduction

The definition of music concept starts from different research fields and its definition angle is different. At present, the widely accepted definition is as follows: The concept of music is defined as an art category that mainly exists through acoustic vibration, is displayed in time, and causes various emotional reactions and emotional experiences through human auditory organs [1, 2]. Music is a kind of flowing art form. In the process of listening and appreciating, music cannot stay and freeze. It is an emotional experience that depends on the audience's instantaneous perception and capture. In addition, from the perspective of people's subjective feelings, music affects people's hearing through the sound effect, and then the audience makes a judgment on this kind of hearing, is happy, sad, thinking, or sad, and then brings an impact on people's intuition and other feelings, and even affects people's feelings and thoughts. Marxism holds that everything is interrelated and complementary with other things except for its own independence, and music is the same [3, 4]. In the analysis and research of music, music cannot be independent but should be combined with related things for analysis, which plays an important role in our comprehensive and in-depth understanding of music. For example, music cognition can be linked to dance, music has a supportive effect on dance, and plays a role as icing on the cake. Music and poetry can also be linked to form a more comprehensive understanding of the art form of rhythm through the common ground between the two. Music and drama can also be combined effectively, and the plot can be developed with ups and downs through the graceful and passionate role of music, so as to foil the inner emotions of the characters.

Different instruments have different timbre characteristics. The basic timbre characteristics of musical instruments mainly depend on the material, shape, sound mode, and overtone characteristics of musical instruments. Musical instruments with different materials, shapes, and sound principles have greatly different overtones produced by sound waves when playing, which is caused by different physical vibration characteristics of different materials, and this is the reason why each musical instrument has its own unique timbre [5, 6]. Erhu's sound is mellow and beautiful, bright and lyrical, deep and graceful. Erhu not only uses old rosewood or small leaf rosewood production but also useful ebony, ebony, gloomy wood, gold nanmu, and other wood production, most of these wood density is higher, texture is relatively hard, with good deformation and vibration resistance and other physical characteristics. The density of old rosewood and ebony is generally smaller than that of wood such as lobular rosewood, so the sound of Erhu made of old rosewood is generally bright, full, and thick, while the sound of Erhu made of lobular rosewood will appear louder and more concentrated. The sound principle of Erhu is to use a bow made of bamboo and horsetail to pull the bow hairs and rub the string to make it vibrate. At the same time, the effective string length is changed by changing fingers and handles by pressing the string with the left hand, thus changing the frequency of string vibration and the overtones produced. Because the wood used by the luthiers is different, each luthier has his own experience in making the instrument. The timbre of the Erhu instruments is also different, just as no two people in the world have the same voice, which belongs to the personality characteristics of the timbre of the vocalizing body [7, 8]. But, we can clearly distinguish between heard voices or Erhu because of voice sound material and other factors, such as voice way of overtones that generate vibration, that is common in tone color, also has the common characteristic. In this article, we discuss the Urheen timbre features, which is based on the Urheen timbre of common features.

Health emphasizes the physical, mental, and social performance of the individual. Health specifically includes two contents, the first is the normal operation of the body viscera, normal development of the body shape, uniform body shape, all body organs, and systems have normal physiological functions and can be engaged in normal labor. This is also a basic requirement for human health. Second, the pointer is more resistant to disease and has a better level of physical performance and physical strength. In modern life, great changes have taken place in people's concept of health. The World Health Organization has added connotation to the definition of health, emphasizing that people should have mental health and good social adaptability, and anti-frustration ability. Health can be discussed in stages, adolescents, vigorous, and thriving health. In adulthood, when the internal organs function properly and the mind is calm and energetic, health is considered. Old age period can live a normal life, modest peace is health. To sum up, it refers to the various functions and organs of the human body that have good function operation, energetic, but also have a better ability to adapt to society. Health mainly refers to the physical ability of a normal person to adapt to the environment for a long period of time [9, 10]. The disease mainly refers to present symptoms of physical dysfunction, or mental and psychological problems.

Music is a way of expressing human emotions. Music can improve people's ability to appreciate, feel and experience beauty, stimulate people's interest in learning, and contribute to the improvement of comprehensive artistic accomplishment. Music can also adjust people's mood so that people can relax, relieve physical and mental, reduce anxiety, improve sleep, and even can be used for auxiliary medical treatment. Music therapy has been rising since the 1950s. After many scientists and medical workers summarize and experiment in research and clinical practice, music therapy has gradually become an independent scientific discipline. In recent decades, it has developed rapidly in various countries around the world and formed modern music therapy. Modern music therapy has realized the comprehensive application of music, medicine, psychology, and other disciplines, and focuses on the treatment of patients under the interaction of various disciplines. However, the research on music therapy in China started late, mainly rising in the late 1970s. After that, music therapy began to explore and learn from some mature experiences and methods of music therapy in China, and was widely used and practiced in clinical practice, so that music therapy could be vigorously developed and promoted. The therapeutic function of music does not mean that music can play a radical role in the treatment of disease, but through the role of music plays a supplementary role in the treatment of disease. The mechanism of music therapy is based on the stimulation of music so that patients can receive this stimulation from the physiological and psychological perspective, and then form a certain influence. Music is a kind of sound wave with rhythm. In the process of listening to music, people are stimulated by sound waves, which will make them feel physically and mentally. Music of these unique charms is just right to stimulate the listener, so as to adjust and improve the function of human body. From the perspective of psychological analysis, through the role of music can stimulate the nervous system, to achieve the comfort of the human visual and auditory system and sensory system, and then relieve psychological pressure and bad emotions so that the psychological positive effect and guidance [11, 12].

In addition to the basic timbre of the instrument itself, the player's manipulation also has a very important influence on the timbre of the instrument, which is the emotional timbre. The same Erhu can produce different timbre in different hands, which is mainly caused by the differences in techniques of different players when playing the instrument. The author believes that there are mainly two links that play a decisive role in the influence of techniques on timbre. The first is that the performer presupposes timbre from the aesthetic point of view, and the second is to realize the presupposes of timbre by using techniques of left and right hands. Both are indispensable. Everyone has the most perfect timbre in his mind, so when playing musical instruments, due to different aesthetic pursuits, the preset standards for timbre are not the same. When it comes to the actual control of techniques, because everyone has different skills and techniques, the difference in timbre may be greater. The influence of techniques on Erhu timbre is mainly reflected in the left-hand techniques. Right-hand technique and special technique are three aspects [13, 14]. The left-hand technique in Erhu performance generally influences the timbre quality, timbre thickness, and timbre tension by changing the string angle of the left-hand finger, the area of the string and the strength of the string, etc. When the left-hand press produced the change of the angle, which in turn has changed the finger touch area, and according to string dynamics change, these a few respects to determine whether the finger to the string vibration filter completely, whether to change the fingers below for effective vibration chord vibration quality and characteristics, finally formed left-hand techniques on Erhu effect.

The first thing you need to do in playing is to establish a feeling. Only when you have a feeling first can the player have content to express and the desire to express what you want. If the performance does not conform to what I think, the performer will try to achieve the effect to be made, driving the performer to constantly practice and improve their performance. This is the importance of the sense of quantity. However, the abovementioned definitions are abstract feelings, which cannot be described in specific words. In the early stage of performance, the performance is only performed through some accumulated perceptual experience. However, these experiences may be blind, random, unreliable, and unscientific, which cannot stand the objective test and may even affect the performance effect. Therefore, if you want to achieve more accurate performance, you must analyze it and listen to whether the actual performance effect meets your expectations. Then what is quantitative analysis? Quantitative analysis is to express ambiguous feelings through data or concrete images. Volume, for example, is determined by decibels, above which is noise. So these are the numbers that give us a clear idea. The basic skills of Erhu are like kneading strings. Everyone knows the basic skills of kneading strings. But when it comes to the music, how to choose the kneading strings, the frequency of kneading strings, the speed, and slowness of kneading strings, and even the specific kneading can achieve the feeling to be expressed. What kind of speed is chosen to express the mood of a piece of music? These need to be quantified analysis, some of the rhythm and beat, we can use the metronome to fix, that for some abstract string kneading, more specific frequency these need us to do different effects in practice, can be compared [15, 16].

## 2. Related Work

Public health-related theories are mainly divided into three aspects: extension-construction theory, affective dynamic model, and neuropsychological theory affecting cognition. The theory of expansion and construction of positive emotions is a highly influential theory in the field of positive emotion research. It was proposed by von Dawans et al. on the basis of further expanding previous studies. It is used to explain the evolutionary adaptive value of positive emotional experience and to clarify the mechanism of positive emotions promoting individual happiness and realizing individual growth. Expanding function and constructing function are the core part of the model. The model holds that positive emotions can expand the scope of individual's immediate thinking and action, including the expansion of individual's cognition and behavior [17, 18]. That is to say, if an individual is interested in something, he or she will take cognitive actions of paying attention to and exploring it and actively acquire experience conducive to the realization of the goal. In the process, new ideas, experiences, and behaviors greatly expand thinking and action. As for the constructive function, the model believes that positive emotions can help individuals construct lasting personal resources, including physical, intellectual, psychological, and social relationships, and thus bring sustainable benefits to individuals. The constructive function is realized on the basis of expansion. In a word, the model emphasizes that positive emotions can expand individual thinking and actions to construct lasting personal resources for individuals, and form a virtuous cycle.

According to the emotional dynamic model of public health proposed by Zautra et al, positive emotions play a pivotal role in goal adaptation. Under normal circumstances, positive emotions and negative emotions affect each other, relatively independent, but if adversity, under the condition of positive emotions will likely too stressful events caused by inhibition of negative emotions play a role, namely, positive emotions buffer stress response of the negative event, the individual's mental health promotion role. In conclusion, this model mainly shows that positive emotions can buffer and inhibit the psychological effects of negative emotions, and then improve subjective well-being and promote personal growth. Neuropsychological theory approaches public health from a biological perspective. According to this model, positive emotions have a cognitive promoting effect, mediated by dopamine. There is evidence that there may be an optimum level for dopamine to mediate positive emotion in cognition. In fact, when comparing induced moderate positive emotions with neutral emotions, not only did dopamine levels increase in various brain regions but there were also significant increases in peripheral blood circulation, such as serum dopamine levels. This is conducive to the agility of thinking and logical improvement [19,20]. This model can be used to understand that public health can promote problem-solving and decision-making, that is, improve the efficiency of problem-solving and the accuracy of decision-making. In conclusion, this model provides strong biological support for other related theories of positive emotions.

As an important birthplace of music therapy, our ancient wisdom has summed up the experience of exploring the mysteries of life with five tones. Through the use of music to cure disease, the impact on human physical and mental health is often found in China's long history. Classical music has a broad sense and narrow sense, here refers to the broad sense of classical music, its creation technique is strict and orderly, elegant and gorgeous style, beautiful and smooth melody, giving people a feeling of relaxed and refreshing. Studies have shown that classical music has a good effect on improving physical and mental health, especially in healing physical and mental trauma. With the development of the times, new ideas emerge in an endless stream, and the pursuit of music creation is becoming more and more free. Modern music is the product of the times, seeking new techniques and new musical language to express oneself and vent their inner feelings. Data suggest that regular exposure to baroque music can help improve physical and mental health and even regulate and alleviate psychogenic diseases. It can be proved that classical music can not only have a good impact on people's physical and mental health but also help children's intelligence [21, 22].

Music therapy has been developing in clinical practice for more than 40 years and has become a very important research subject in the current stage. A number of research results show that both classical music and modern music have an impact on people's physical and mental health, and there are certain differences. Music affects the brain in a way that controls the emotional connection between music and the sound we hear, a study suggests. Singing can be carried out anytime and anywhere. Compared with musical instruments, dancing and other forms of music are also easier to learn. Therefore, it is more loved by people. For the vast majority of people who love singing, most of them love life, their hearts are full of sunshine, and singing enables them to learn the correct use of breath, increase lung capacity, and improve their physical condition. Pop music has a variety of structures, broad content, easy to understand, easy to accept, sincere emotion, and changeable style, which is loved and received by the majority of the people. Usually, pop song of drawn from real life, belongs to the type of songs for young and old, has their positive side, but part of modern pop music songs and lyrics are so thief, too decadent, negative, and moaning whinge bags song causes to people's physical and mental health development has a certain negative effect. Especially for people of different stages, the lyrics of popular songs do not really consider people's psychological acceptance, which causes people in the lower age stage to have wrong cognition in such lyrics. Now under the influence of pop music [23, 24], people's physical and mental health development issues need to be attentive, due to the wider range of a part of popular songs, the interval between spans is also relatively large, sometimes even need to be a hysterical scream, this kind of situation will be a certain adverse influence on the elderly and children. Therefore, people of different ages should be discriminated against when choosing pop music. They should not go with the flow, otherwise, they will misjudge their outlook on life and values.

The art of Erhu timbre expression requires three points. First of all, it accurately reflects the mood or color that the music or performer wants to express through timbre. Gestalt psychology shows that the relationship between the movement of things or the morphological structure of things is similar to human physiology or psychology. In other words, the heterogeneous homomorphic relationship in music art is expressed as the ups and downs of music and the fluctuation of people's thoughts and emotions. No matter what genre the composer uses, from classical music to modern music to avant-garde music, composers of different eras have different pursuits, and performers have the same way of using timbre to express musical mood or color. Secondly, it is necessary to accurately reflect the characteristics of vocalization of Erhu performance through timbre. In addition, the Erhu has no quality, no phase, no fingerboard, and the bow can freely express the importance of music, so the characteristics of the Erhu sound can be clearly displayed. Finally, when timbre has an accurate expression of mood and phonological characteristics, we can enter into the use of timbre to establish a musical image. A musical image can be a scene, a character, or a spirit. The change of timbre and people's inner activities can produce an isomorphic relationship, which can make people connect the emotions conveyed by timbre with the scenes they see in daily life, so as to form the imagination of music image [25, 26].

As an instrument good at imitating the sound cavity, Erhu timbre plays an important role in the process of shaping the sound cavity. First of all, timbre can express the mood of the voice cavity. Secondly, timbre can show the image of sound cavity. When must show women spoke characteristic, can use faster speed and smaller bow you touch pressure as far as possible use WaiXian to emit bright, mellow tone. The expression of men spoke characteristics, you can use a larger bow pressure and the touch area, try to use the string a vigorous, hale timbre, to reflect the music image. Finally, timbre can reflect the style of sound cavity. When shaping the sound cavity, the style of different sound cavities is largely reflected by timbre. When Erhu imitates the singing style of Jiangnan local opera, its timbre should be gentle and clear. The Erhu can easily connect and change notes during the operation of the cavity [27, 28]. When the cavity changes, the Erhu can imitate the operation of the cavity by relying on its no-substance, no-phase strings to play the notes without trace. It is precise because the Erhu can imitate the vocal cavity with a high degree of reduction through the manipulation of timbre and techniques that in many local operas, the Erhu and other huqin instruments play a very important role in the accompaniment or the tone preservation of the opera. The melodies of many Erhu songs are characterized by tonality. In particular, many Erhu works based on local operas and folk music have the vocal performance of different local operas and folk music, coupled with a bow that can flexibly reflect priorities and cadences. We can use the combination of various techniques to get rich timbre and tone changes, so as to meet the needs of the performer in the performance of sonication.

From a physical point of view, Erhu performance is nothing more than a series of continuous sound waves in nature, the smallest unit of which is sound. The sounds used in Erhu performance are a series of articulation units with fixed frequency or pitch and duration. The music is produced in the development of long-term musical practice and consists of a series of different sounds. Then, according to certain rules, all kinds of sound columns form a specific system, which is used to express musical ideas and shape musical images. There are four kinds of sound attributes: high and low, strong and weak, length and timbre. The pitch is determined by the number of times the object vibrates within a certain period of time. If you vibrate more, you get a higher tone. If you vibrate less, you get a lower tone. The range of audio that the average human ear can hear is about 30–16,000 Hertz. The length of the sound is determined by the duration of the vibration. The long duration of the vibration is long and the short duration of the vibration is short. We can find out the characteristics of the timbre from the process of Erhu performance. Erhu performance is an activity in which the performer makes the Erhu sound by operating the Erhu. The sound generated is transmitted to the listener's ear by sound waves, and the extraction of sound characteristics can be completed at any stage in this process [29, 30]. Each stage is the player's manipulation of the instrument, the instrument's formation of sound waves, and the listener's hearing of sound. In the process of Erhu forming sound waves, the source of sampling is the sound waveform, that is, the recording of the amplitude of sound waves within a certain sampling frequency. It is necessary to carry out various analyses of the audio data and finally get the required musical features, which involves a lot of pattern recognition knowledge. Pattern recognition is still a hot research topic and there are still many areas to be improved. The pattern recognition of sound is widely used in speech recognition and has some research achievements in music feature extraction [29, 31].

It can be seen from the literature that before deep learning was introduced into the field of Erhu performance evaluation, the research focus was mainly on feature extraction and classifier selection. With open source music data sets, Erhu genre classification research in the field of heat rising, deep learning early application in the field of music genre classification, is used as a classifier have been proposed, most of the research work is to extract the Erhu attribute expression feature extraction, and ignoring the depth of learning ability of the model. As it is difficult to define the correlation attribute between extracted features and Erhu performance effect, performance effect evaluation based on these underlying features is difficult to ensure the classification effect. The selection of feature sets has a great impact on Erhu performance effect evaluation, and traditional evaluation algorithms are difficult to deal with large-scale music works. In order to solve the abovementioned problems of limited Erhu performance evaluation, deep learning music genre classification algorithms began to emerge. Chen et al. [32] improved the structure of the convolutional neural network by increasing the network depth and improving the feature extraction effect of the network model through a repeated convolutional layer and its corresponding pooling layer. Luke et al. [33] took the original audio signal of music generated by Mayer filtering as the input of the model, realized the learning of music attribute features and genre attribution determination through the convolutional recurrent neural network, and compared the genre classification performance of DCNN with different convolutional kernels at different scales and in different convolutional modes. In 2021, Dhaka et al. [34] proposed a deep CNN model, which combined channel attention mechanism and one-dimensional residual convolution to effectively extract features from audio spectrograms after data enhancement, so as to realize evaluation of Erhu performance effect. Therefore, the evaluation of Erhu performance effect in this topic is based on the extraction of Erhu timbre based on deep learning technology. Hence, the main contributions of this paper are

1. This paper is the first to introduce the DDPSO method into the application field of the analysis of Erhu performance
2. The research in this paper not only has good theoretical results but also has great potential application value

## 3. The Proposed Analysis of Erhu Performance Effect in Public Health Method

### 3.1. CNN Model Introduction

This paper uses the feature extraction model of CNN (Convolutional neural network), the advantage of this method lies in its deep learning architecture, which can extract music features very well and can solve the problem of Analysis of Erhu performance effect in public health music works, and the structure of CNN is shown in Figure 1. Since the CNN model has been relatively mature, its theoretical knowledge and practical application can be easily found in the existing literature. Therefore, limited to the reasons of length, this paper will not be repeated here. The key technologies of data processing represented by CNN model can no longer efficiently and timely process the data generated by Erhu performance effect in public health music works. In order to handle this problem, the optimized CNN model is introduced in this paper.

The function of the convolution layer is shown as follows:

(1) $$\begin{array}{c} {\text{CONV}}_{\left(ij\right)}=\sum_{i}^{m-1}\sum_{j}^{n-1}u_{ij}\times w+b\left(i=1,2\ldots m-1;j=1,2\ldots n-1\right), \end{array}$$

where *u*_*ij*_ is the input image, *m* and *n* are the sizes of the input image, and thus the value range of *m* and *n* are the whole set of real numbers. *w* is the size, and *b* is the bias constant. *CONV*(*ij*) is the output after convolution.

Then, the description of sigmoid function is as follows:

(2) $$\begin{array}{c} f\left(x\right)=\frac{1}{1+e^{-x}}. \end{array}$$

The Tanh function is as

(3) $$\begin{array}{c} f\left(x\right)=\frac{e^{x}-e^{-x}}{e^{x}+e^{-x}}. \end{array}$$

The ReLu function is as

(4) $$\begin{array}{c} f\left(x\right)=\max\left(0,x\right). \end{array}$$

The Leaky-ReLu function can solve the abovementioned problem.

(5) $$\begin{array}{c} f\left(x\right)=\left\{\begin{array}{cc} x, & x\geq 0,\\ \alpha x, & x<0. \end{array}\right. \end{array}$$

Thus, the corresponding equations of Sig and Tanh are as follows:

(6) $$\begin{array}{c} \left\{\begin{array}{c} sig\left(x\right)=\frac{1}{1+\exp\left(-x\right)},\\ \tanh\left(x\right)=\frac{\exp\left(x\right)-\exp\left(-x\right)}{\exp\left(x\right)+\exp\left(-x\right)}, \end{array}\right.\\ h_{w,b}\left(x_{i}\right)=\left[\begin{array}{c} p\left(y_{i}=1|x_{i};w,b\right)\\ p\left(y_{i}=2|x_{i};w,b\right)\\ p\left(y_{i}=3|x_{i};w,b\right)\\ \cdots \\ p\left(y_{i}=n|x_{i};w,b\right) \end{array}\right]=\frac{1}{\sum_{j=1}^{n}e^{w_{j}x_{i}+b_{j}}}\left[\begin{array}{c} e^{w_{1}x_{i}+b_{1}}\\ e^{w_{2}x_{i}+b_{2}}\\ e^{w_{3}x_{i}+b_{3}}\\ \cdots \\ e^{w_{n}x_{i}+b_{n}} \end{array}\right]. \end{array}$$

Finally, the cross entropy (CE) formula is as follows.

(7) $$\begin{array}{c} \mathrm{loss}=-\frac{1}{m}\sum_{j=1}^{m}\sum_{i=1}^{n}y_{ji}\log\left({\hat{y}}_{ji}\right). \end{array}$$

The error calculated from the CE function is shown as follows:

(8) $$\begin{array}{c} \theta ≔\theta -\alpha \frac{\partial }{\partial \theta }J\left(\theta \right). \end{array}$$

The description of a typical Adam optimizer is given as

(9) $$\begin{array}{c} m_{t}=\beta_{1}m_{t-1}+\left(1-\beta_{1}\right)g_{t},\\ v_{t}=\beta_{2}v_{t-1}+\left(1-\beta_{2}\right)g_{t}^{2}. \end{array}$$

Therefore, the gradient descent update process is shown as

(10) $$\begin{array}{c} \theta_{t+1}=\theta_{t}-\frac{\alpha }{\sqrt{v_{t}+\epsilon }}m_{t}. \end{array}$$

### 3.2. Improved Optimization Algorithm

Since conventional CNN is prone to local optimality. Particle swarm optimization (PSO) is simple and easy to solve, but it is prone to local extreme points, low accuracy, slow convergence, and stagnation. In this section, the differential perturbation is introduced into the PSO to form the differential perturbation particle swarm optimization (DPPSO) algorithm, which makes use of the advantages of fast convergence speed and good global performance of difference, overcomes the shortcomings of low precision and local optimal caused by the use of PSO, and builds an optimized CNN model. It is worth noting that the improved PSO algorithm proposed in this paper is used to optimize the parameters of CNN model, such as the number of hidden layers, number of nodes, and so on, which is to achieve the best analysis of Erhu performance effect in public health music works model performance in this paper The multi-objective optimization model is given as follows:

(11) $$\begin{array}{c} \begin{array}{cc} \min & f_{1}\left(x_{1},x_{2}\right),\\ \max & f_{2}\left(x_{1},x_{2}\right),\\ \text{s.t.} & \begin{array}{c} p_{1}<g_{1}\left(x_{1},x_{2}\right)<q_{1},\\ p_{2}<g_{2}\left(x_{1},x_{2}\right)<q_{2},\\ p_{3}<g_{3}\left(x_{1},x_{2}\right)<q_{3},\\ p_{4}<g_{4}\left(x_{1},x_{2}\right)<q_{4}, \end{array} \end{array}\\ 120<x_{1}<180,\\ 120<x_{2}<180, \end{array}$$

where *f*_1_ represents energy consumption target, *f*_2_ represents the output target. *g*_1_, *g*_2_, *g*_3_, *g*_4_ represent the packaging quality of 4 indicators: crushing strength, wear strength, drop strength, and compressive strength, respectively.

### 3.3. The Framework of the Proposed Method

Although the structure of the optimized CNN model can be designed by many different methods, the model design selected for this paper is given as in Figure 2, mainly because it can achieve the best analysis of Erhu performance effect under this setting. Based on the abovementioned discussions, the optimized deep neural network and its application in analysis of Erhu performance effect in public health music works are shown in Figure 2. In conclusion, it can be seen from the results of Figure 2, it includes the original data, the data preprocessing, the model training and testing, and the performance evaluation, which means that the proposed method has reasonable flow and rigorous logic.

## 4. Experimental Results and Analysis

### 4.1. Data Collection and Experimental Environment

Due to the lack of parallel data sets of the same musical work performed in different styles, different researchers mostly use different data sets constructed by themselves to conduct relevant music style conversion experiments. It is generally believed that music of the same genre has the same style. This paper collects and downloads Erhu music of marked genre from relevant music platforms on the Internet to construct a performance style data set. In the GTZAN dataset, the duration of each piece of Erhu music data is about 20 seconds, and each genre has 1000 pieces of music data, with a total of 10,000 pieces. In this experiment, 70% of them are taken as training sets, 15% as verification sets, and 15% as test sets. Relevant information on Erhu music is analyzed.

The setting of learning rate is very important to the convergence effect of network model. In deep CNN, when the learning rate is too large, the model is difficult to reach the convergence state, and continuous oscillation will occur within the adjacent range of the minimum value. When the learning rate is too small, the time required for the model to reach the convergence state will be greatly increased. After many comparisons and experimental verification, the model learning rate in this paper is set to 0.01. In this paper, the accuracy of genre classification and the loss function value of feature extraction is used as the performance evaluation indexes of the model. Genre classification accuracy refers to the accuracy of the model to classify music genres. The loss function of feature extraction is calculated by the cross entropy function which is more suitable for multi-classification problems. The network model and comparative experiment designed in this paper are constructed based on TensorFlow framework in a Python environment. The details are shown in Figure 3. Although there are many ways to deal with the structure of the convolution layer and pooling layer, the structure in this paper is the best result obtained according to the test data. In addition, as the most common activation function, ReLu function is also selected in this paper, and a two-layer full connection layer is set in the designed CNN model.

### 4.2. Experimental Results Analysis

In order to illustrate the influence of iteration times on model training, the validation set was tested with a learning rate of 0.01 and iteration times of 50. The changes in classification accuracy and loss of the model are shown in Figure 4. As can be seen from the figure, the model classification accuracy increases first and then tends to be stable as the number of iterations increases. And when the accuracy of genre classification tends to be stable, the number of iterations can be approximately 10. The loss function value of feature extraction decreases first and then tends to be stable with the increase of iteration number. According to the figure, the number of iterations when the loss function value of feature extraction tends to be stable can be approximately 8.

By analyzing the experimental results of the model, the classification effect of the model on music genres has reached a stable state when the iteration is 10. At this time, the loss function value of model feature extraction tends to be stable. In order to ensure the effectiveness of model training and the training efficiency of the model, 10 times were selected as the number of training iterations of the model in this paper. It is worth noting that the left ordinate in Figure 4 is the range of the loss function, while the right ordinate in Figure 4 is the range of the accuracy, so their ranges are different. In this paper, the coordinate axes of these two scopes are plotted together in Figure 4.

Furthermore, the loss curve function of different feature extraction ways (which is shown in Figure 5). As can be seen from Figure 5, after feature enhancement of the audio spectrum, the value of model loss function also decreases. According to the results of features-enhanced ablation experiment, after filtering the original audio signals, dimensionality reduction can effectively improve the expression of Erhu genre characteristics, and thus improve the accuracy of Erhu genre classification. Moreover, the reduction of the loss function value of feature extraction indicates that the proposed model has a good convergence speed and loss reduction effect, which verifies the advanced and effectiveness of filtering on the improvement of the feature extraction effect of Erhu. Based on the analysis of experimental data, the model can effectively learn the differences in the expression of musical characteristics, such as tone strength and rhythm, to achieve a good judgment of the music of different schools. However, in the feature extraction of the music genre, it is easy to lose part of the information of audio signals and reduce the correlation between audio signals. Therefore, two different methods are selected for feature extraction of original Erhu audio signals, and the expression effect of music rhythm and genre features is enhanced. It is worth noting that the two feature extraction methods in Figure 5 are the conventional CNN model and the optimized CNN model, respectively. Obviously, the feature extraction of the optimized CNN model is better than that of the unoptimized CNN.

In addition, Figure 6 shows the distribution of Erhu features with different frequencies in three-dimensional space (where different colors represent Erhu features with different frequencies). As can be seen from the figure, the feature distribution of the first three low frequencies has a great difference, showing a normal distribution trend basically. However, purple features with high frequency have a gentle distribution area and a smaller amplitude than the previous features. But the wavelength range of all four frequencies is roughly the same. In a real design the appearance, though, there are many different types of features. However, only 4 kinds of most representative design styles (different frequencies) are selected here to verify the validity of the proposed method.

After that, in order to verify the distribution of performance characteristics of Erhu with different tones at the same frequency.  Figure 7 shows the features classification of high, middle, and low tones. As can be seen from the figure, no matter what frequency characteristics (subject to normal distribution or not). In most coordinate dimensions, this method can obtain better results of Erhu performance feature extraction and classification. The results show that the method presented in this paper can distinguish the performance characteristics of different frequencies and different tones of the Erhu well, so as to have a good performance evaluation performance of the Erhu. It is worth noting that Figure 7 shows the features classification of high, middle, and low tones. Hence, the horizontal and vertical coordinates of Figure 7 are dimensionless values, that is, they have no units.

Finally, Figure 8 presents the distribution of Erhu performance characteristics in different positions. As can be seen from the figure, it is affected by wind speed. However, features of Erhu performance were extracted in different positions of Erhu performance, and the distribution of these features was relatively uniform, which indicated that the proposed method could extract more performance features, so as to describe the performance effect of Erhu in a more comprehensive way.

## 5. Conclusion

The most important thing in Erhu performance is feeling, and feeling will be expressed purposefully. Performance evaluation is one of the important performance techniques. It is an important factor supporting Erhu performance, so the quantitative analysis of performance effect is to achieve better performance effect, make a qualitative change, and accumulate in the long term to achieve the possibility of quantitative change. Therefore, it is important to emphasize its importance in daily practice. The more accurate the analysis, the more effective the practice will be.

On the basis of relevant research, this paper proposes the research of Erhu performance evaluation based on an optimized deep learning model. The CNN model based on PSO optimization is used to extract the sequence of Erhu feature vectors and analyze the distribution of different features, so as to better evaluate the performance of Erhu. The research in this paper has not only theoretical significance but also potential application value. Although the method in this paper has achieved good performance, it is still a lightweight deep model. In the face of big data scenarios, depth-based resource optimization methods will be the focus of future research.

## Figures and Tables

**Figure 1:** The schematic diagram of CNN.

**Figure 2:** The model structure diagram of the proposed method.

**Figure 3:** The CNN structure designed in this paper.

**Figure 4:** The changes in classification accuracy and loss of the model.

**Figure 5:** Loss curve function of different feature extraction ways.

**Figure 6:** Distribution of erhu features with different frequencies.

**Figure 7:** The features classification of high, middle, and low tones.

**Figure 8:** Distribution of erhu performance characteristics in different positions.

## Data Availability

The experimental data used to support the findings of this study are available from the corresponding author upon request.
